# Comprehensive Evaluation of BIM Calculation Quantity in Domestic Construction Engineering Based on Fuzzy Comprehensive Evaluation

This article has been retracted.

**DOI:** 10.1155/2021/3292376

**Published:** 2021-12-31

**Authors:** Yi Deng, Ziyuan Rao, Ling Cai

**Affiliations:** ^1^School of Architecture and Urban Planning, Guangzhou University, Guangzhou 510006, Guangdong, China; ^2^Guangdong Provincial Institute of Cultural Relics and Archaeology, Guangzhou 510075, Guangdong, China

## Abstract

Nowadays, with the leap-forward development of computer technology and the transformation of information technology management concepts, China's construction industry is quietly entering the era of refined management. Accurate estimation and cost control have become among the key considerations of the construction industry. For the calculation of engineering quantity, there are already many software devices that can be used for the calculation of engineering structure quantity, which means that the incorrect operation of personnel has been reduced to some extent, improving the work efficiency and measurement accuracy. The purpose of this paper is to solve the problems of computational missing, computational errors, inefficiency, data loss, and repetitive system in traditional computing based on the advantages of BIM computing system, which provide a reliable basis for cost forecasting and control. At the same time, using BMI calculation system to solve the problem of steel reinforcement in construction engineering, as well as the use of personnel, the existing calculation software still needs a lot of time and energy. We proposed a comprehensive evaluation study of reinforcement calculation in domestic construction engineering BIM calculation system based on a fuzzy comprehensive evaluation. This paper first summarizes the BIM calculation system of construction engineering, uses fuzzy comprehensive evaluation system as an important evaluation index system in domestic construction engineering BIM calculation system, through the judgment of various factors affecting the actual effect of the calculation system, and uses the fuzzy evaluation system combined with a case to demonstrate the superiority of the proposed research. Therefore, through the above research and experiments, it is concluded that the research method of this paper solves many problems in the process of engineering structure reinforcement calculation and provides a good reference method for the establishment of comprehensive evaluation system of reinforcement calculation, as well as providing an effective validation for the widespread use of BIM technology in the construction industry. Finally, it is also beneficial for users to comprehensively evaluate the BIM calculation system of the construction industry and provide a basic reference condition for different industries to use and choose BIM calculation systems.

## 1. Introduction

With the rapid development of information technology, building informatization has received more and more attention. As an important tool for building informatization, BIM has received strong government support and implementation in Britain, United States, Japan, South Korea, and other countries. With the pace of building informatization, we actively join the ranks of research and application of BIM technology [1]. As a new management concept, BIM integrates and applies project information through building information systems, provides an information exchange platform for project participants, and improves the management, decision-making, and service levels of project participants [2]. Scholars and companies actively responded to the call of the country, conducted a lot of research on the application of BIM technology in various stages of construction engineering, and developed different BIM calculation systems for the realization of BIM calculation methods [3].

However, in practical applications, the BIM calculation system has not played the expected advantages, and the problems of low engineering calculation efficiency and difficulty in information accumulation and sharing still exist [4]. It even brought a series of new problems, such as the difficulty of reusing design information, inconsistent system standards, and high thresholds for user operations, which severely affected the enthusiasm for the application of BIM calculations in China and hindered the promotion and implementation of BIM technology [5]. Therefore, it is necessary to conduct a comprehensive evaluation study on the BIM calculation system of construction engineering, establish an effective BIM calculation system evaluation index system and comprehensive evaluation system, provide reliable references and suggestions for the selection and improvement of the BIM calculation system, and promote BIM calculation system promotion and application, and fuzzy comprehensive evaluation is an available good method. Fuzzy comprehensive evaluation has the characteristics of clear results and strong systematicness. It can better solve the fuzzy and difficult quantification problems and is suitable for the solution of various uncertain problems. Therefore, it can improve the shortcomings of the current BIM calculation comprehensive evaluation [6].

The effective application of BIM technology in engineering calculation, solving traditional calculation problems, improving computational efficiency and quality, and providing reliable data support for cost control is one of the best methods in engineering management [7]. The comprehensive evaluation and research of the domestic BIM computing system will promote the promotion and application of BIM calculation [8]. The purpose of this paper is to study the BIM calculation theory, discuss the connotation and characteristics of the BIM calculation system, define the BIM calculation system and analyze its functional requirements, and provide a theoretical basis for the comprehensive evaluation of the BIM calculation system in domestic construction projects [9]. We understand the research status of BIM calculation system at home and abroad, and based on the research of relevant literature and standards, establish a BIM calculation system and comprehensive evaluation system for domestic construction projects of evaluation index system, and calculate the amount addition system for comprehensive evaluation. Through the actual project case study of the indicators affecting the application of BIM computing system in domestic construction projects, the comprehensive evaluation results are verified to provide a basis for the selection of BIM computing systems in the future [10]. Countries have vigorously promoted the application boom of BIM in construction, but the functions of various BIM calculation systems are still immature, and there are incompatible problems between system data, which has hit the application enthusiasm of BIM in construction. Many enterprises have begun to hold conservative attitude, promoting BIM technology and information construction [11]. Secondly, the establishment of the domestic BIM calculation system evaluation index system and comprehensive evaluation system will help users understand the advantages and disadvantages of each BIM calculation system and help users quickly select the appropriate BIM calculation system to promote the development of domestic BIM calculations [12]. Finally, the comprehensive evaluation and case analysis computing system can help see the development status of BIM computing system in China, understand the actual needs of BIM's defect computing system and users, promote the full realization of BIM computing value, and promote the development of information construction [13].

This article is based on the synthesis of BIM technology and computing software. By studying the current situation of BIM technology and computing software in the current market, the problems of BIM technology and reinforcement calculation software in application are clarified, and the importance of BIM technology in domestic construction engineering is put forward. On the basis of learning BIM technology, the application value of BIM technology in the calculation of construction industry is analyzed and summarized. Combined with the above problems, the importance of fuzzy evaluation in the domestic construction engineering BIM calculation system is determined. By reading a large number of references, it can be found that the domestic construction industry has not played its due role in the BIM calculation system, and there are still many problems in the construction industry, resulting in less research on the comprehensive evaluation system of BIM calculation. The user chooses the BIM calculation system, lacking an effective evaluation index system and a comprehensive evaluation system. This paper is aimed at the above problems, that is, an in-depth study of comprehensive evaluation theory, determining the construction principles, construction methods, and indicators selection methods of BIM computing system index system. By comparing and analyzing the engineering calculation methods of different stages of workflow and information transmission process, the functional scope of BIM computing system is defined in different periods, and the domestic BIM computing system establishes the target decomposition method and expert of evaluation index system through literature research methods. The investigation method points out that BIM is of great significance for the comprehensive evaluation of the construction engineering quantity calculation system.

This paper is divided into five parts. The first section mainly introduces the purpose and significance of the BIM calculation system in the domestic construction industry and provides a basic evaluation index system for the domestic construction engineering BIM calculation system based on fuzzy comprehensive evaluation. Make a corresponding statement. The second section mainly introduces the basic concept of BIM calculation system and the role and connection of fuzzy comprehensive evaluation system in the domestic construction industry and finally explains the research methods and research details of this paper. The third section mainly introduces the relevant settings of the experiment, including the experimental environment design, the source of the experimental data, and specific steps of the experiment. The fourth section is the experimental discussion of this article, mainly summarizing the detailed experimental details. The fifth section concludes that the research of this paper is summarized on the basis of a large number of experiments, and the problems existing in this paper and the direction of the next research are elaborated.

## 2. Proposed Method

### 2.1. Related Work

#### 2.1.1. Research Status of BIM Calculation System and Comprehensive Evaluation Method

At present, the research on BIM technology is relatively more, but the research on introducing fuzzy evaluation system into BIM calculation system in construction industry is relatively less [14]. In the BIM manual, Biswas TK analyzes the system creation method that supports project planning control, summarizes the benefits of the system application to the project, and gives BIM a lot of advice on many projects and provides a lot of advice [15]. Comprehensive evaluation refers to the establishment of a corresponding mathematical system to integrate the results of multiple individual evaluation indicators into a comprehensive and comprehensive evaluation result. In the 1980s, the “efficiency coefficient method” led to the comprehensive evaluation of statistics applied to the comprehensive evaluation of social and environmental economic benefits in various industries. The application of comprehensive evaluation has been diversified [16]. At present, the comprehensive evaluation method has matured and applied widely in modern times. Commonly used comprehensive evaluation methods include analytic hierarchy process, grey comprehensive evaluation method, artificial neural network evaluation method, data envelopment analysis method, and fuzzy comprehensive evaluation method [17].

#### 2.1.2. Domestic Research Status of BIM Calculation System in Construction Industry

Zhang J believes that the core idea of BIM computing system is integrated design and construction, analyzes the functions of visual simulation, communication, and collaborative BIM computing system, and proposes CAD-based system method and BIM technology from the perspective of system integration [18, 19]. Wei and Zhang first analyzed the characteristics of the construction project and the introduction of the system, expounded the impact of the construction process simulation, analysis, and construction process management functions, and considered that the system application can be played in the schedule and cost management. Its role improves project management level and production efficiency. The four-dimensional building information system technology defined in the memorandum of understanding is the research object. It introduces and summarizes the existing BIM technology and system technology research results and then proposes a feasible system building plan according to the actual construction management and information integration requirements, thus achieving schedule management. To some extent, based on the Revit platform [20], there are few domestic researches on the application of BIM technology in schedule management. Biswas has further explored the application status of BIM technology in the planning and control of domestic construction industry projects and further explored the scheduling and BIM technology in the schedule control [21]. Wang found the cause of the problem based on the analysis of the problems in the progress management of the engineering project and then compared the difference between the traditional management technology advancement and the advantages of the BIM-based 4D technology demonstration application BIM-based 4D construction. Simulation technology is in progress management [22].

### 2.2. Overview of Fuzzy Comprehensive Evaluation Method

The measures to evaluate the comprehensive benefits of construction projects based on artificially set standards, the results of which contain people's subjective consciousness, are inaccurate. Therefore, in the evaluation process, the fuzzy relationship comprehensive principle is applied to quantify the comprehensive benefit factors of construction engineering measures with unclear boundaries and difficult evaluation [23]. Therefore, a comprehensive evaluation system based on fuzzy mathematics is established to objectively reflect the control effect of construction engineering measures and provide an objective basis for the application of construction engineering measures [24].

The fuzzy weight vector *A* and the fuzzy relation matrix *R* are synthesized by a reasonable fuzzy synthesis operator, and the fuzzy comprehensive evaluation result vector *B* of each evaluated object is calculated. The commonly used fuzzy synthesis operators include *M* (∧, ∨), *M* (·, ∨), *M* (∧, ⊕) and *M* (·, ⊕). The synthetic operator system of fuzzy comprehensive evaluation in this study is *M* (·, ⊕). Weighted average type can be expressed as

(1) $$\begin{array}{c} B=WR=\left[w_{1},w_{2},...,w_{m}\right]=\left(b_{1},b_{2},...,b_{m}\right). \end{array}$$

The evaluation result vector *B* is a description of the degree of membership of each level of the evaluation object. The self-assessment result is a fuzzy vector and cannot be directly used for sorting and selection [25]. The comprehensive analysis results should be used to calculate the comprehensive score of each evaluation object, sorted by size, and select the best order. This paper mainly uses the weighted average principle to process the results and finally determines the relative position of the evaluation objects [26].

#### 2.2.1. Method for Determining Index Weight

The index weight represents the value and relative importance of each inspection index of a tested object in the whole, as well as the quantitative value of the proportion. The methods of determining weights mainly include subjective weighting method and objective weighting method. The subjective weighting method mainly includes the analytic hierarchy process, the Delphi method, and the expert scoring method. The objective weighting method mainly includes the standard deviation method, the entropy weight method, the shadow method, and the coefficient of variation method. In the process of establishing fuzzy comprehensive evaluation system, Delphi and AHP methods are usually used to assign weights to evaluation indicators, but their weight values are highly subjective, and the results of complex problems are less objective. Therefore, this paper chooses the combination of objective weighting method and subjective weighting method to empower qualitative indicators and quantitative indicators [27, 28]. In the objective evaluation method, the shadow method can combine the influence of the indicator change on the weight and the conflict between the indicators. Therefore, this paper considers the use of the AHP method combined with the critic method to determine the index weights.

The importance of each indicator in objective weights is measured by contrast strength and conflict. Let *C*_*j*_ indicate the amount of information in the *j* evaluation indicator; then, *C*_*j*_ can be expressed as

(2) $$\begin{array}{c} C_{j}=\sigma_{j}\overset{n}{\underset{t=1}{\sum }}\left(1-r_{tj}\right),\;j=1,2,\ldots ,m. \end{array}$$

The more obvious the change in *C*_*j*_, the more the corresponding content of the *j* indicator included, which means that the more representative the index, the objective weight *w*_*j*_ of the *j* indicator should be

(3) $$\begin{array}{c} W_{j}=\frac{C_{j}}{\sum_{i=1}^{n}C_{j}},\;j=1,2,\ldots ,m. \end{array}$$

According to certain criteria, each element on the same target layer is compared in pairs to determine the relative importance of each element. After establishing the comparison judgment matrix, it is necessary to further determine the eigenvalue and weight vector and perform consistency check. Only when the consistency test is reasonable can the rationality of the matrix be determined.

The consistency check step includes the following indicators to calculate the consistency indicator CI:

(4) $$\begin{array}{c} \text{CI}=\frac{\lambda_{\max}-n}{n-1}+\frac{\beta_{\text{min}}-\beta }{o-1}*\prod \left(\beta +\lambda \right). \end{array}$$

The larger the CI value, the greater the degree of matrix deviation consistency; the closer the CI to 0, the better the matrix consistency.

According to the random consistency indicator RI, calculate the consistency ratio (CR):

(5) $$\begin{array}{c} \text{CR}=\frac{\text{CI}}{\text{RI}}+\frac{\text{z}u}{eu}*{\left(a_{u}+b_{k}+z_{c}\right)}^{a+bn}, \end{array}$$

where CI is the calculation consistency index, and a, *b* and *z* are constants. When CR > 0.1, the matrix does not meet the consistency requirement, and the construction matrix needs to be regenerated. When CR < 0.1, the matrix consistency is better.

The weighting results of the shading method and the analytic hierarchy process are comprehensively weighted. Objective weights are used to assist subjective weights and improve the accuracy of subjective weights. Combine subjective and objective weights and comprehensively evaluate the results. The comprehensive weight calculation formula is as follows:

(6) $$\begin{array}{c} W_{\text{sum}}=\frac{W_{T}\cdot W_{A}}{{\sum W_{T}\cdot W}_{A}}. \end{array}$$

The composite weight of the target layer is synthesized from top to bottom by the weights of the indicators at all levels, and finally, the combined weights of the lowest level indicators are obtained.

#### 2.2.2. Membership Function

Establish the membership function of each evaluation factor with the object to be evaluated: when the indicator is a quantitative indicator, the evaluation factor is a large-scale function; then,

(7) $$\begin{array}{c} r_{ij}=\left\{\begin{array}{cc} 0, & x<a,\\ {\left(\frac{x-a}{b-a}\right)}^{k}, & a\leq x\leq b,\\ 1, & x>b, \end{array}\right) \end{array}$$

*r*_*ij*_ represents the membership function. When the size of *X* is different, its value and calculation method are also different.

When the evaluation factor is a small function, then

(8) $$\begin{array}{c} r_{ij}=\left\{\begin{array}{cc} 1, & x<a,\\ {\left(\frac{b-a}{b-a}\right)}^{k}, & a\leq x\leq b.\\ 0, & x>b. \end{array}\right) \end{array}$$

When the indicator is a qualitative indicator, the index value is obtained by the hierarchical scoring method, and the membership function selects a linear function. The evaluation factor is a large function; then,

(9) $$\begin{array}{c} r_{ij}=\left\{\begin{array}{cc} 0, & x\leq a,\\ \frac{x-a}{b-a}, & a<x<b,\\ 1, & a<x\leq b,\\ \frac{d-x}{d-c}, & c<x\leq d,\\ 0, & x>d. \end{array}\right) \end{array}$$

When the evaluation factor is a small function, then

(10) $$\begin{array}{c} r_{ij}=\left\{\begin{array}{cc} 0, & x\leq a,\\ \frac{x-a}{b-a}, & a<x\leq b,\\ \frac{c-x}{c-b}, & b<x\leq c,\\ 0, & x>c. \end{array}\right) \end{array}$$

This is a grouping and stratification of multiple evaluation indicators according to the nature of the problem, according to the top level (objective a), the middle level (first-level evaluation index *b*_i_, *i* = 1, 2,…, *m*), and the bottom level (two *A* three-level (or multilevel) evaluation index system arranged in the form of c_ij_, *i* = 1, 2,…, *m*; *j* = 1, 2,…, *n*_*i*_). Then, we build the fuzzy judgment matrix。

To construct the fuzzy evaluation matrix, firstly, the single factor in the hierarchical structure system in Figure 1 needs to be considered. *c*_*ij*_, (*i* = 1, 2,…, *m*; *j* = 1, 2,…, *n*_*i*_) is a single factor evaluation. From the factor bi, (*i* = 1, 2,…, *m*), focusing on the elements of the belonging relationship, *C*_*ij*_ has the membership degree of *a*_*jj*_ to the judgment set *v*_*j*_ (*j* = 1, 2,…, *n*), so that the single factor judgment set of the *j*-th element *C*_*ij*_ under the bigrouping is obtained:

(11) $$\begin{array}{c} d_{m}=\left(d_{n1},d_{n2},\ldots ,d_{nn}\right). \end{array}$$

In this way, the evaluation set of *n*_*j*_ factors constructs an evaluation matrix *D*_*m*_, (*m* = 1, 2,…, *i*); that is, each evaluated object is determined from bi, (*i* = 1, 2,…, *m*). The fuzzy relationship to *C*, that is, the matrix:

(12) $$\begin{array}{c} D_{m}={\left(a_{jj}\right)}_{i_{m}\times i}=\left[\begin{array}{cccc} a11 & a12 & \ldots & {\text{a}1}_{i}\\ a21 & a22 & \ldots & a2_{i}\\ \ldots & \ldots & \ldots & \ldots \\ a_{i_{n}1} & a_{i_{n}2} & \ldots & a_{i_{n}i} \end{array}\right]. \end{array}$$

Specifically, *a*_*jj*_` represents the frequency distribution of the *i* factor *C*_*ij*_ on the *i*`th comment *v*_*j*_ under the bigrouping.

Specific steps are as follows.

First, the optimal matrix *D* needs to be constructed.

(13) $$\begin{array}{c} D={\left(d_{ij}\right)}_{ni\times ni}. \end{array}$$

The optimal matrix *D* is defined as a three-valued matrix (0, 0. 25, 0. 5) on a finite universe *C* = (*c*_1_, *c*_2_,…, *c*_*n*_). Obviously, *D* is a fuzzy complementary matrix.

Secondly, construct the fuzzy consistent judgment matrix *G*.

(14) $$\begin{array}{c} G={\left(g_{ij}\right)}_{ni\times ni}. \end{array}$$

After the optimization table is established, it is converted into a fuzzy consistency matrix. The fuzzy consistent judgment matrix *G* is a multivalued matrix *G*=(*g*_*ij*_)_*ni*×*ni*_ on the finite universe *A* = (*a*_1_, *a*_2_,…, *a*_*n*_) and 0 < *g*_*ij*_ < 1. *G*_*ij*_ shows the relative importance of *a*_*i*_ to *a*_*j*_: if 0 < *g*_*ij*_ < 0. 25, it means that *a*_*j*_ is more important than *a*_*i*_, and the smaller the *g*_*ij*_, the more important the *a*_*j*_ than *a*_*i*_; if *g*_*ij*_ = 0.25, it means that *a*_*i*_ and *a*_*j*_ are equally important; if 0.25 < *g*_*ij*_ < 0.5, it means that *a*_*i*_ is more important than *a*_*j*_, and the larger the *g*_*ij*_, the more important it is.

In the conversion process, the preferred matrix *D*=(*d*_*ij*_)_*ni*×*ni*_ needs to be summed by rows, namely,

(15) $$\begin{array}{c} T_{j}=\overset{n_{j}}{\underset{k=1}{\sum }}e_{jk},\;j=1,2,\ldots ,n_{j}. \end{array}$$

Then,

(16) $$\begin{array}{c} g_{ij}=\frac{t_{i}-t_{j}}{2n_{j}}+0.5. \end{array}$$

The final matrix *G*=(*g*_*ij*_)_*ni*×*ni*_ is the fuzzy consistency matrix 。

Then, calculate the matrix's *G*=(*g*_*ij*_)_*ni*×*ni*_ max. The normalized feature vector is the standard weight set *w*_*i*_^*T*^.

According to the fuzzy judgment matrix *D*_*m*_ established above and the calculated weight set *w*_*i*_^*T*^, the evaluation vector *B*_*j*_ of the second layer is calculated:

(17) $$\begin{array}{c} B_{j}=w_{i}^{T}\times D_{m},\;i=1,2,\ldots ,m. \end{array}$$

Using the results of the hierarchical comprehensive evaluation, the comprehensive evaluation matrix *D* can be obtained. Based on this, the comprehensive evaluation can be obtained. Valence vector:

(18) $$\begin{array}{c} C=w^{t}\times D+\left[\begin{array}{cccc} {\text{e}}_{11} & e_{12} & i & e_{1o}\\ e_{22} & e_{23} & i & e_{2o}\\ n & n & p & n\\ e_{n1} & e_{n2} & i & e_{nn} \end{array}\right]. \end{array}$$

The hierarchical evaluation vector *B*_*j*_ and the comprehensive evaluation vector *C* are, respectively, multiplied by the comment score set V to obtain the evaluation score of each index, and finally the evaluation result is analyzed.

Using logic gate circuit thinking, *P*(*r*_*i*_) is a binary function of yes or no:

(19) $$\begin{array}{c} P\left(r_{i}\right)=P\left(x,y,s_{i}\right)=\left\{\begin{array}{cc} 1, & d\left(s_{i},p\right)\leq R_{s},\\ 0, & \text{other.} \end{array}\right) \end{array}$$

As long as any node in the node set covers grid point *q*(*m*, *n*), it is said that grid point *q*(*m*, *n*) is covered by node set *C*. Probability *P*(*x*, *y*, *C*) represents the probability that grid point *q*(*m*, *n*) is covered by the current working node set *C*; then,

(20) $$\begin{array}{c} P\left(x,y,C\right)=P\left(\overset{n}{\underset{i=1}{\cup }}r_{i}\right)+q\left(\overset{o}{\underset{u=1}{\cup }}e_{u}\right). \end{array}$$

Extending formula (20), we get

(21) $$\begin{array}{c} P\left(\overset{n}{\underset{i=1}{\cup }}r_{i}\right)=1-\overset{n}{\underset{i=1}{∐}}\left(1-P\left(x,y,s_{i}\right)\right). \end{array}$$

The sum of the grid area covered by the working node set *C* is the sum of the grid area covered by each node in the node set, denoted as Area(*C*); then,

(22) $$\begin{array}{c} \text{Area}\left(C\right)=\int_{0}^{x}\int_{0}^{y}P\left(x,y,C\right)\text{d}x\text{d}y. \end{array}$$

If there are too many grid points, a large number of distance calculations will be performed according to the above method, and a large part of the nodes in these calculations have exceeded their sensing radius, so it is a meaningless calculation. Excessive calculations will prolong the solution time. Therefore, the algorithm needs to be improved appropriately.

In the wireless sensor network, a binary vector *X*=(*a*_1_, *a*_2_,…, *a*_*N*_) is used to indicate whether each node is working or shutting down. *a*_*i*_=0 means that the node is off, and *a*_*i*_=1 means that the node is on. *f*_1_(*X*) and *f*_2_(*X*) respectively represent network coverage and node utilization. Their calculation formula is

(23) $$\begin{array}{c} f_{1}\left(X\right)=\frac{\text{Area}\left(C\right)}{\left(m\times n\right)},\\ f_{2}\left(X\right)=\overset{N}{\underset{i=1}{\sum }}\frac{a_{i}}{N}+\overset{\text{m}}{\underset{u=1}{\sum }}\frac{x_{u}}{o}. \end{array}$$

The goal of the wireless sensor network coverage optimization problem is to maximize network coverage while minimizing node utilization. Therefore, this problem needs to consider the combination of network coverage and node utilization at the same time. Solving such problems is usually to construct a linear combination of goals through weighting.

So, the center position of point *X*_*i*_ is

(24) $$\begin{array}{c} \text{center}\left(X_{i}\right)=\underset{j=1,i-1,\ldots ,i-n}{\text{most}}\left(a_{j1},a_{j2},\ldots ,a_{jN}\right). \end{array}$$

In the actual application process, in the relevant system entropy theory, the entropy value tends to be larger, which means that the higher the degree of integration of chaos, the less information it carries. On the contrary, if the information entropy is smaller, then it will carry more information. The entropy method uses the meaning of entropy to calculate the entropy value of the discrete degree of the data to be evaluated. The specific calculation process is as follows:

(25) $$\begin{array}{c} a=\left(\begin{array}{ccc} a_{11} & \cdots & a_{1o}\\ \vdots & \cdots & \vdots \\ a_{n1} & \cdots & a_{no} \end{array}\right)+\left(\begin{array}{ccc} b_{10} & \cdots & b_{up}\\ \vdots & \cdots & \vdots \\ b_{o1} & \cdots & b_{op} \end{array}\right)+\left(\begin{array}{ccc} c_{12} & \cdots & c_{vm}\\ \vdots & \cdots & \vdots \\ c_{z1} & \cdots & c_{e0} \end{array}\right). \end{array}$$

Among them, *a*_*uk*_ is used to represent the value of the evaluation index, *u* is the sample, and *k* is the evaluation index.

(26) $$\begin{array}{c} f_{k}=-g\overset{n}{\underset{u=1}{\sum }}b_{uk}\text{out }b_{uk}+\overset{o}{\underset{m=1}{\sum }}z_{uk}x_{uk},\\ g=\frac{1}{\text{out }n}\min\left(1,\overset{n}{\underset{u=1}{\sum }}d_{u}e_{uk}\right),\;k=1,2,i,o,\\ y_{k}=\overset{n}{\underset{u=1}{\sum }}d_{u}e_{uk}+\overset{n}{\underset{u=1}{\vee }}\left(d_{u}\wedge e_{uk}\right). \end{array}$$

Among them, *g* is a constant. Its value directly affects the size of the weight. The greater the *g*, the greater the *f*_*k*_ value. The smaller the *g*, the smaller the *f*_*k*_ value. The greater the importance of the evaluation, the greater the weight.

(27) $$\begin{array}{c} d_{k}=\frac{w_{k}}{\sum_{u=1}^{n}w_{k}}+\frac{d_{g}}{\sum_{v=1}^{o}d_{g}}+\frac{f_{h}}{\sum_{m=1}^{p}f_{h}}. \end{array}$$

The weight of the *k*-th indicator is *w*_*k*_=1 − *f*_*k*_.

In summary, the algorithm is optimized. We can start the experiment.

### 2.3. Objectives and Principles of Fuzzy Comprehensive Evaluation of BIM Calculation System

There are many influencing factors in the BIM calculation system, including technical aspects, policy aspects, standards, users, and industry environment. Each influencing factor will have a different nature and varying degree of impact on the BIM calculation system. To ensure the rationality and effectiveness of the evaluation index system, the following principles need to be followed when constructing the evaluation index system of the BIM calculation system:

1. Target: according to the results, the fuzzy comprehensive evaluation measures with better performance are selected to provide a certain basis for the optimization of fuzzy comprehensive evaluation measures. Based on the basis, reduce the blindness of fuzzy comprehensive evaluation measures in the application practice process, make it play a better role, and provide a reliable basis for the application and promotion of fuzzy comprehensive evaluation measures.
2. Principle: there are many factors that reflect the comprehensive effectiveness of fuzzy comprehensive evaluation measures. It is extremely important to select the evaluation factors with sensitivity, representativeness, and rationality among many evaluation factors. Therefore, when establishing a comprehensive evaluation system for comprehensive evaluation of fuzzy comprehensive evaluation measures, it should follow the purpose, theory, objectivity, independence, and operability.
3. Purpose: the establishment of any system is for a certain purpose. The land use in urban areas is complex and different from the underlying surface of the basin. Therefore, the factors selected in the evaluation must reflect the comprehensive effectiveness of fuzzy comprehensive evaluation measures. Theoretically, the theory is the basis and guiding basis for the evaluation method and evaluation criteria in the establishment of the rating system, and it is also a prerequisite for reliable and reasonable evaluation results.
4. Objectivity: subjective judgment should be abandoned in the process of system establishment, and objective usability should be maintained to make the evaluation results more realistic. Independence and comprehensiveness: in the process of selection, the evaluation indicators should not only maintain the independence of each indicator, but also cooperate with other indicators to reflect the comprehensiveness of the whole system. Operability: when selecting evaluation indicators, it should be as easy as possible to ensure that the indicators are easy to obtain, with strong reliability and measurability, as well as ease of analysis.

The structure of the Internet of Things system can be divided into the perception layer to obtain data, the network layer to transmit information, and preprocessing. The application layer provides services to users, a total of three layers. The corresponding layer needs to be completed through the relevant technology of each layer. Tasks and services, sensors, controllers, machines, people, and things are connected in new ways by using communication technologies such as local network or Internet to form a network of people and things, and things and things, so as to realize informatization, remote management and control, and intelligence. The related architecture diagram is shown in Figure 2.

The underlying structure is shown in Figure 3.

Among the Internet of Things technology, RFID technology and ZigBee technology are important components, and they have been widely used and studied in various fields. RFID technology is a kind of automatic identification technology. It carries out noncontact two-way data communication through radio frequency and uses radio frequency to read and write recording media, so as to achieve the purpose of identification target and data exchange; ZigBee technology is a short-range, low-power wireless communication technology. Compared with traditional tags, Table 1 shows the technical advantages of RFID over traditional tags.

The topological structure used by the system is different, the corresponding system is different, and the parameter settings of each node in the network are also different.  Table 2 compares the characteristics of three different ZigBee topologies.

## 3. Experiments

### 3.1. Data Source

The total construction area of the resettlement area is about 200,000 square meters and is divided into two parts. The total construction area of the first phase is about 100,720 square meters, of which the total floor area of the ground is about 72006 square meters, and the total underground construction area is about 28,713 square meters. The second batch has a total construction area of 102,222 square meters, 70876 square meters above ground, and 31,346 square meters underground. It consists of 5 high-rise residential buildings (up to 26 floors), 1 multiple floor kindergarten, and 1 multiple floor community service room.

This article is aimed at #3, the second section of residential buildings in the resettlement area. The three buildings cover an area of 12,938.55 square meters, of which the above-ground construction area is 11,580.76 square meters, and the underground construction area is 1357.79 square meters. The total height of the building is 77.2 meters, 26 floors above ground, 3 underground floors, raft foundation, and frame shear wall structure.

The collected BIM data is imported into the rebar list for data preprocessing and system. Finish the steel sheet data. The necessity of the preparation of the steel bar list is analyzed, and the whole preparation work is divided into two parts: CAD table data extraction and steel bar table format conversion.

### 3.2. Experimental Steps

Because the comprehensive evaluation of the BIM calculation system is highly professional, in order to ensure the reliability and validity of the weights of the indicators, this paper constructs a judgment matrix by issuing questionnaires to 35 experts with rich BIM knowledge and work experience. MATLAB software is programmed to calculate the maximum eigenvalue of the judgment matrix and its corresponding eigenvector and check the consistency of the calculation results. Finally, the weighted average of the index weights of each expert is performed to obtain the comprehensive weight of each index, and the index is sorted by importance. Judgment matrix is the name of linear algebra tool matrix used in decision-making. In decision analysis, the matrix constructed to compare factors is one factor in horizontal and vertical dimensions, and the matrix element is the decision value of one dimension element corresponding to another element. Construct a judgment matrix, calculate weights, and perform consistency checks in Table 3.

A1: the judgment matrix for the second-level indicators of computing ability is shown in Table 4.

A2: calculate the judgment matrix of the secondary index of quality is shown in Table 5.

A3: judgment matrix of calculation efficiency secondary index is shown in Table 6.

A4 with attributes and capabilities is shown in Table 7.

The A5 report function is shown in Table 8.

BIM calculation system management and application calculation results first-level index weight calculation are shown in Table 9.

BIM calculation system management and application calculation results secondary index weight calculation are shown in Table 10.

“G” and “L” BIM calculation systems each have 100 copies. In order to ensure the reliability of the questionnaire, questionnaires that have been exposed to the BIM calculation system for less than one year are removed, and finally there are 87 valid questionnaires remaining in the “G” BIM calculation system.  Table 11 is the educational level of the G and L survey subjects.

“G” BIM measurement system survey target unit category is shown in Table 12.

“L” BIM measurement system survey target unit category is shown in Table 13.

“H” BIM measurement system survey target unit category is shown in Table 14.

“I” BIM is the same, so we will not repeat it here.

## 4. Discussion

### 4.1. Comprehensive Analysis of Project Progress Based on BIM

1. No matter how detailed the plan is, it is impossible to foresee all the possibilities, and there will still be deviations during the execution of the project plan. Tracking project schedules and controlling project changes are the main tasks of the implementation phase. Take necessary corrective measures to ensure that the project progresses steadily within the deadline and budget. In the process of project implementation, the analysis of resources is mainly based on reviewing the differences in working hours and checking whether the resource allocation is too much or insufficient. Based on the resource configuration table, resource histogram, or resource curve combined with the Gantt chart tracking view, the resource allocation status and usage status of the selected time period are displayed, and the resource allocation problem is discovered in time, as shown in resource allocation (Table 15).
2. After inputting the actual progress information in the system, in order to avoid the problems caused by the deviation, the project needs to constantly adjust the objectives, such as adjusting the allocation of manpower or resources and adjusting the construction time, and take appropriate measures to solve the problems. Project completion time, total cost, and resource allocation often deviate from the original plan, so it is necessary to take corresponding measures to make the project development more in line with the original plan. Resource allocation and budgeting costs need to be adjusted. The experimental results are shown in Figure 4.

It can be seen from the figure that the amount error is large, and the maximum value is 25%, but the total error is small. At Q3, the three errors are consistent and reach the minimum value (Figure 6).

### 4.2. BIM Calculation System Fuzzy Comprehensive Evaluation Results

1. In order to study the factors that can cause some adverse effects on the BIM metering system, the “G” and “L” BIM computing systems are used to simulate the actual situation of #3, and the calculation results are managed and applied. “G” BIM system and “L” BIM system 3# residential building are shown in Figure 5.
2. Through the application of the “G” and “L” BIM computing systems, it is found that both have good visual computing functions, can operate the components in three-dimensional state, clearly display the position and overlapping relationship of complex components, and make the calculation work more vivid and intuitive. In addition, the two BIM computing systems can also display 3D between components for easy inspection and discovery of system errors, as shown in Figure 4. In contrast, the deduction information between the components displayed by the “G” BIM calculation system is more detailed, and the detailed calculation process of the engineering quantities of the parts intersecting the components can be clearly seen, and the partial 3D deduction map can also be displayed.

Introduce the technical parameters of F-SAR as shown in Figure 7.

The classification performance of the ensemble learning methods used by the two satellites is compared with the results obtained by SVM classification. The values in the columns of the different methods indicate the classification accuracy of different data sets. The experimental results are shown in Figure 8.

Figure 9 shows the simulation results of different TMI splitting ratios.

Combining with OpenGL graphics technology, this article uses simulation-generated TLE data to carry out comparative experiments. Real-time simulation of the target needs to be rendered and output after position calculation. Therefore, the statistics of the experiment include two parts: position calculation time and rendering time.  Figure 10 shows the comparison of CPU and GPU time consumption below 30,000 orders of magnitude.

The specific results are shown in Figure 11.

In order to test the delay time and resource consumption of the server in the process of obtaining the data released by the device side and obtaining the data on the user side when the load of the server is gradually increasing, in this test, the server side is deployed on the third-generation platform based on the Linux operating system. The performance test network structure is shown in Figure 12.

This is a star topology, with the middle control center as the midpoint, connecting satellites, servers, and other components, so as to test the network performance.

The test result is shown in Figure 13.

Then, we have done satisfaction statistics on the system designed in this article. In the overall analysis of satisfaction with the new system, the questionnaire uses a Likert 5-level scale, with a total of 1, 2, 3, 4, and 5 ratings, which are very dissatisfied, dissatisfied, fair, satisfied, and very satisfied. The lowest score is 1 point, and the highest score is 5 points. The higher the score, the higher the satisfaction level, and vice versa. Use SPSS24.0 software to analyze the average satisfaction data of the recovered new system. The specific distribution is shown in Figure 14.

The comparison between uniform random distribution LKNN and DV-Hop is shown in Figure 15.

The comparison between C-shaped random distribution LKNN and DV-Hop is shown in Figure 16.

## 5. Conclusions

Through the analysis, it can be seen that the calculation amount of the “G” BIM calculation system and the “L” BIM visual calculation quantity function also has certain limitations, such as only one type of component on the single floor, 3D editor; this restricts the user system creation idea to some extent. Two BIMs are proposed to measure the visual function of the system and further improve the user's autonomy, allowing the user to select and operate multiple floors and several work pieces at the same time. Two plus one: in general, the visual function of the computing system enriches the calculation process, makes the information more accurate, comprehensive, and intuitive, reduces the data analysis and error propagation in the process, and improves the BIM calculation system. Operational: to a certain extent, improve the credibility of the calculation results. The “G” and “L” BIM calculation systems have a high conversion rate for CAD drawings. As long as the CAD drawings are identified and converted according to the import rules provided by the system, and attention is paid to the details, the main components can be accurately imported. For individual components that cannot be converted, manual adjustments are required.

BIM calculation improves the calculation accuracy and efficiency and realizes the collaborative sharing of calculation results and the accumulation of computational experience. In order to study the BIM application computing system obstacles, help users better use the BIM calculation system, BIM calculation of the number of construction engineering system comprehensive evaluation of this paper, through the development of BIM calculation system and the status quo at home and abroad, and BIM. Applying the calculation quantity and obstruction, system analysis, and comprehensive evaluation, the concept of comprehensive evaluation of BIM calculation amount of domestic construction projects is proposed. On the basis of computational theory, comprehensively evaluate and analyze the workflow and information transfer process of different stages of calculation methods, combined with the development of 3D system technology, computational quantity system functional requirements analysis, and point out that BIM is a measurement system and should include both system management and application computing and application. The literature evaluation method, target decomposition method, and expert investigation method are used to select and revise the system evaluation index of BIM calculation. The factors that can be used to study the BIM calculations hinder the application of the domestic construction engineering and the actual needs of the users, as well as the selection and BIM calculation system.

In summary, with the increase of construction engineering activities, the importance of comprehensive evaluation of BIM calculation system has become increasingly prominent. In order to improve the accuracy of project supervision and evaluation, and to ensure the objective and fair evaluation of the evaluation, it is necessary to improve the fuzzy comprehensive evaluation method. Applying the improved fuzzy comprehensive evaluation method to the comprehensive evaluation of BIM calculation system can not only ensure the comprehensiveness of information, but also promote the orderly conduct of supervision and evaluation and provide reliable theoretical support for the establishment of evaluation. In addition, Chinese scholars should explore and improve the index system in depth, establish a reasonable fuzzy evaluation system of entropy weight, and give full play to the application advantages of the improved fuzzy comprehensive evaluation method, which is of great significance for the smooth construction of construction projects. Therefore, China's construction engineering supervision unit should use this as a reference to improve the utilization rate of fuzzy comprehensive evaluation methods.

## Figures and Tables

**Figure 1:** Resource allocation map.

**Figure 2:** Internet of things technology architecture chart.

**Figure 3:** Schematic diagram of the underlying structure.

**Figure 4:** Rendering resource renderings.

**Figure 5:** 3# residential building standard layer “G” BIM calculation system.

**Figure 6:** Effect of two BIM calculation systems on fasteners.

**Figure 7:** F-SAR technical parameters.

**Figure 8:** Algorithm performance comparison based on different data sets.

**Figure 9:** Simulation results of different TMI splitting ratios.

**Figure 10:** Comparison of CPU and GPU time consumption below 30,000 orders of magnitude.

**Figure 11:** Comparison of CPU and GPU time.

**Figure 12:** Performance test network structure.

**Figure 13:** Performance test results.

**Figure 14:** Overall situation of satisfaction degree.

**Figure 15:** The comparison between uniform random distribution LKNN and DV-Hop.

**Figure 16:** The comparison between C-Shaped random distribution LKNN and DV-Hop.

**Table 1:** Traditional tag and RFID tag features contrast.

Feature	Traditional label	RFID label	Data sources	Reliability (%)
Antifouling ability	Paper version, easy to break and be contaminated	The label uses a chip to store information, so it is resistant to strong pollution capacity	IEE6.0	96.5

Reusable	Not recyclable, because all the information, once printed, cannot be changed	The content can be modified, added or delete and other operations, so it can be recycled	CER221	94.8

Recognition speed	Read the information of one tag at a time at close range	Using the principle of electromagnetic coupling, it can be long-distance Read multiple tags at once	DAP101	96.8

Capacity	Can store up to 3000 characters	The amount of stored data is dozens of times that of barcodes	EFG660	99.5

Penetrability	No penetration communication	Can penetrate wood, metal, plastic, etc. The advantage of nontransparent material, can penetrate communication	CDE3.0	68.7

Safety	Data content can be arbitrarily smeared and tampered with	Data content realizes password through encoding, protection, internal information is not easy to be forged and changed	INT250	89.9

**Table 2:** Characteristics of ZigBee network topology.

Type	Typical characteristics	Credibility (%)	Safety (0-1)
Star topology	Including a coordinator and multiple terminal devices, the network structure is easy to maintain and has good real-time performance, but there is only one data transmission path, the coordinator may affect the transmission of network data, which can be used in data transmission small scene	99.6	0.9

Cluster topology	The structure is complex, and the network can be transmitted in a multi-hop form; it has the performance characteristics of self-organization and self-coordination	99.5	0.89

Mesh topology	The information is sent in time, the stability is good, and the storage space required is large. At the same time, the cost of maintaining the network is more than more expensive, it can be used in places where the designed ZigBee network is more complicated	99.7	0.96

**Table 3:** BIM calculation system amount first-level index judgment matrix.

*α*	A1	A2	A3	A4	A5	*W*
A1	1	1	3	3	5	0.3424
A2	1	1	3	3	5	0.3424
A3	1/3	1/3	1	1	3	0.1298
A4	1/3	1/3	1	1	3	0.1298
A5	1/5	1/5	1/3	1/3	1	0.0556

**Table 4:** A1: the judgment matrix for the second-level indicators of computing ability.

A1	A11	A12	A13	A14	*W*
A11	1	1/3	3	3	0.2828
A12	3	1	3	3	0.4732
A13	1/3	1/3	1	1	0.1220
A14	1/3	1/3	1	1	0.1220

**Table 5:** A2: calculation of the judgment matrix of the secondary index of quality.

A2	A21	A22	A23	*W*
A21	1	3	3	0.6000
A22	1/3	1	1	0.2000
A23	1/3	1	1	0.2000

**Table 6:** A3: judgment matrix of calculation efficiency secondary index.

A3	A31	A32	*W*
A31	1	3	0.7500
A32	1/3	1	0.2500
A33	1/2	0.8	0.4500
A34	1/4	0.5	0.1500

**Table 7:** A4: judgment matrix with secondary index of attribute ability.

A4	A41	A42	A43	*W*
A41	1	5	1	0.4546
A42	1/5	1	1/5	0.0909
A43	1	5	1	0.4545

**Table 8:** A5: report function secondary index judgment matrix.

A5	A51	A52	A53	*W*
A51	1	3	3	0.6000
A52	1/3	1	1	0.2000
A53	1/3	1	1	0.2000

**Table 9:** BIM calculation system management and application calculation results first-level index judgment matrix.

*β*	B1	B2	B3	B4	*W*
B1	1	1	3	3	0.3750
B2	1	1	3	3	0.3750
B3	1/3	1/3	1	1	0.1250
B4	1/3	1/3	1	1	0.1250

**Table 10:** BIM calculation system management and application calculation results secondary index judgment matrix.

B2	B21	B22	B23	*W*
B21	1	1	1	0.3333
B22	1	1	1	0.3333
B23	1	1	1	0.3333

**Table 11:** BIM calculation system survey object education level.

	“G” BIM (%)	“L” BIM (%)	“H” BIM (%)	“I” BIM (%)
Master's degree	33.33	44.05	54.31	61.25
Undergraduate	60.92	54.76	58.21	59.84
College degree and below	5.75	1.19	2.93	3.11

**Table 12:** “G” BIM measurement system survey target unit category.

	Institutions of higher learning (%)	Construction unit (%)	Construction unit (%)	Consulting service unit (%)	Cost consulting unit (%)	Others (%)
Value	26.44	24.14	19.54	5.57	18.39	5.75
Mean	24.12	20.63	20.16	4.37	17.54	6.15
Even	25.55	21.45	21.22	5.66	18.17	6.33

**Table 13:** “L” BIM measurement system survey target unit category.

	Institutions of higher learning (%)	Construction unit (%)	Construction unit (%)	Consulting service unit (%)	Cost consulting unit (%)	Others (%)
Value	20.24	19.05	46.43	7.14	2.38	4.74
Middle	21.45	18.79	45.01	6.89	3.31	3.85
Average	22.56	19.99	45.02	7.35	2.95	3.78

**Table 14:** “L” BIM measurement system survey target unit category.

	Institutions of higher learning (%)	Construction unit (%)	Construction unit (%)	Consulting service unit (%)	Cost consulting unit (%)	Others (%)
Value	41.6	36.1	28.5	6.14	3.52	5.78
Max	26.8	21.56	26.84	5.89	2.89	6.78
min	24.56	23.74	27.89	6.99	4.43	4.44

**Table 15:** Resource allocation table.

	Total	Cumulative	Amount
Actual quantity	23	34	66
Quantity still needed	45.37	79.45	47
Over-allocation	45.34	79.34	89.34
Limited quantity	10	10	10

## Data Availability

This article does not cover data research. No data were used to support this study.
